# The impact of economic and political reforms on environmental performance in developing countries

This article has been retracted.

**DOI:** 10.1371/journal.pone.0257631

**Published:** 2021-10-05

**Authors:** Jin Zhao, Ghulam Rasool Madni

**Affiliations:** 1 School of Finance, Shanghai Lixin University of Accounting and Finance, Shanghai, China; 2 Department of Economics and Business Administration, Division of Management and Administrative Science, University of Education, Lahore, Pakistan; Universidad Nacional Autonoma de Nicaragua Leon, NICARAGUA

## Abstract

The humans of modern society are enjoying the luxuries and comforts today but future generations will be facing a more polluted environment and scarcity of natural resources. So the effects of global warming and climatic changes are a major policy concern nowadays around the world. The majority of the literature treats the Carbon Dioxide emissions as an indicator of environmental deterioration but this paper considers the environmental performance index as an indicator of environment. This paper addresses the role of institutional reforms for environmental performance that is hardly discussed in the earlier literature. It is argued that a novel approach of institutional reforms can provide some useful insights for environmental performance in developing countries. There is wide agreement that institutional quality is crucial for economic sustainability but rarely focused to explore the impacts of institutional reforms on environmental performance. The institutional reforms are generally divided into two categories; economic and political reforms. This paper investigated the impact of each category of institutional reforms for environmental performance by using panel data of 122 developing economies for a period of 1996–2020. Difference in differences technique is applied to determine the impact of each category of reforms on the environment. It is found that economic and political reforms significantly contribute to protecting the environment in developing countries, and it will be a good policy option to reform the economic and political institutions to preserve the environment in these countries along with sustainable development.

## 1. Introduction

Environmental protection is one of the biggest problems confronted by humanity at present. Ever increase in population and per capita consumption are depleting the natural resources as well as the environment. Moreover, industrialization, urban concentration and modern forms of agricultural methods are polluting the water, soil and air resources all over the world. The natural environment is becoming hazardous and toxic for the endurance of future populations. The rising emissions of greenhouse gases (GHG) are affecting the blue planet and estimations of “United States Development Authority” and “Organization for Economic Cooperation and Development” reveal the rise in earth temperature by 2 centigrade by the end of 2050. It will have more adverse effects on the earth. Global warming is causing melting glaciers and polar ice with two to three times higher as compared with last century while loss of biodiversity is unpredictable and unforeseen. There is a sharp increase in saline soils by 50% up to 2050, resulting in land deterioration in every country.

Environmental challenges are not specific to geo boundaries, and steps taken by a single country alone are not sufficient to protect the global environment. The green and sustainable economy requires a basic transition of social, economic, and energy systems. Environmental and economic policies are important for the green economy along with improvement of prevailing institutions for effective implementation and monitoring of policies [1]. Environmental involvement are essential economic policies eventually employed in a wider institutional setting [2]. To achieve the objectives of environmental policies, the political process directing policy adoption plays a central role in conjunction with the nature of institutions, social and cultural discourse, industrial structure, distribution of resources [3–5]. While the role of institutional quality and governance is overlooked by the quantitative models [6].

The theoretical foundations for institutional quality in the context of environment protection highlight that stronger and efficient institutions lead to better policy adoption and its outcomes. The enforcement of rules by the government reduces the level of environmental degradation. The political institutional quality is usually represented by Polity IV that shows the democratic or autocratic regimes in a country. The democratic countries have better control on environmental performance while resources are concentrated to few people in autocratic countries so the cost of public goods lie on those capturing these resources. When democracies are mature then interest of individual groups merge into common interest since gains from environmental performance decrease. Moreover, democratic countries have stronger commitments to international environmental agreements. The inefficient institutional quality leads to sub-optimal use of available resources. The corrupt officials allow the activities which damage the natural environment.

To improve the institutional quality in any country, there is dire need to reform the existing institutions. Institutional reforms are efforts to alter the regulations and constraints influencing human’s dealings. It may be considered as formation of actions, their implementation, management of crisis and way of interaction with other entities. Institutions and their reforms are at the main front of literature as well as in the vision of policy makers since the past two decades. IMF, World Bank, and other donor organizations are of great interest now to reform institutions for financial and other forms of support [7–16]. New institutional economics has two broader sets of literature; impact of institutions on economic activities and effect of institutional reform on economic variables. The set of former literature can be divided into further two sets; first emphasizes the impact of different measures of economic institutions [7–9, 11–13, 17–19] while second describes the effects of political institutions [20]. Similarly, impacts of institutional reforms are highlighted in numerous studies but their role for environmental performance is little elaborated [21–29]. The theoretical reason for institutional reforms in the perspective of the environment is given by the public good feature. Private agents remain unable to calculate the pollution costs due to allied externalities, generating the reason for government interference [30]. Related questions comprise how the nature and different forms of institutional reforms affect environmental performance. In this perspective, Dasgupta and Mäler [31] are of the view that reforming the political institutions are somewhat persuasive in assuring environmental performance. Deacon [32] highlights that democracy is more likely to assure higher levels of environmental quality, arguing that autocracy provides such public goods inefficiently because resources are controlled by a small group. These findings are supported by numerous studies [33–35]. Democracy has a negative relationship with CO_2_ emissions, water pollution, land deterioration, and deforestation rates [36, 37].

Economic institutions are laws, regulations, and policies regulating the relationships among economic agents in an economy along with restrictions on agents to connect in agreed economic transactions. These institutions ensure the incentive mechanism and structure, affecting technology level, investment in humans and physical capital, and way of production. The central objective of economic institutions is minimizing transaction costs. The rule of law, policies affecting consumption and production, property rights, and regulatory quality are examples of economic institutions. While political institutions are constraints concerned to organizing the polity, how power is controlled, legitimated, constituted, redistributed, and exercised.

Stern [38] highlighted many factors causing the deterioration of the natural environment but economic actors amend their attitudes in context of institutional requirements. Democracy is another institutional factor contributing significantly to preserve the environment [39, 40]. Mukherjee and Chakrabotry [41] found a positive relationship among environmental quality, socio-political and socio-economic factors. They are of the view that institutional quality, good governance and level of democracy cause the advancement or decline of environmental performance. It is explained that efficient rules in a society cause to reduce pollution, arguing that strong rules turn “Environmental Kuznets Curve” (EKC) at lower per capita income [42]. Culas [43] found that contract enforcement by government reduces the deforestation rate, while Bhattarai and Hammig [44] highlighted that civil liberty and political rights also cause in reduction deforestation rate.

Environmental protection is one of the gigantic challenges and major focused area for governments, policy makers, researchers, scholars, and academicians involving countries, communities, and individuals around the globe. Environmental sustainability is the major approach contrary to the background of the population growth of humans and uncontrolled exploitation of the natural environment by human activities. The major interest of modern society is that humans are enjoying the luxuries and comforts today but future generations will be facing a more polluted environment and scarcity of natural resources. It is our responsibility to maintain the earth in a self-sustainable manner ensuring equal opportunities to our future generation along with other living species cohabiting with us.

Environmental protection requires a fundamental transformation of economic, political, social and energy systems. The targeted policies will be helpful in steering the transition but it requires more improvement in institutional quality to ensure the implementation of policies and effective monitoring. Environmental policies are ultimately implemented by institutions prevailing in a country. The objectives of environmental policies are dependent on the political process having the ability of policy adoption along with underlying institutions, industrial structure and distribution of power and resources. It is obvious that the importance of institutional reforms cannot be negated if the challenges related to environmental performance are to be tackled on the global, regional, national, and local level. There are numerous factors examined by earlier studies of environmental performance and institutional quality but the relationship between variables of institutional reforms and environmental performance have to be discussed extensively. Institutional reforms are rarely elaborated in earlier macroeconomic analysis of environmental quality. The research question is devised as the impact of institutional reforms on environmental performance in developing countries. The economies without institutional reforms to protect the environment have been heavily criticized over the years. The question is whether or not institutional reforms could positively affect environmental performance. Thus, it is the intention of this study to explore the impact of reforms on environmental performance. To address this issue, a panel of 122 developing countries is selected by considering their economic, political, and environmental indicators to test the relation between institutional reforms and environment. The broad objectives of the study are to explore the impacts of political and economic reforms on environmental performance in developing countries, investigating the interaction effects of each type of reforms. So data is used for 122 developing economies covering the period of 1996–2020 while the difference in difference (DID) regression approach is used for data analysis.

After introduction, section II explains the methodology of the paper. The next section comprises details of data and its sources then empirical findings and discussion are explained in the section IV. Section V concludes the paper.

## 2. Methodology

This study used the difference in difference (DID) technique for estimation that is suitable to determine the effect of pre and post reforms experiences. This approach calculates the outcomes for two time periods of treated and control groups. The pre reform groups are considered as “control” while post reform groups are considered as “treated”. If the same units in a group are present in each period, then the average obtained in the control group is deducted from mean value of treatment group to resolve biasedness issues. To find the effect of reforms on environmental performance, it can be expressed as;

$$EP_{it}={ϴ}_{i}+{ϴ}_{t}+ϴREF_{it}+{ϴ}_{1}Z_{it}+\epsilon_{it}$$ (1)

where **EP** is environmental performance, ϴ _***i***_ is “time invariant impact” unique to individual *i*, ϴ _***t***_ expresses the common impact in time period *t* for all individuals, REF is institutional reform, Z represents control variables and ***ϵ***_***it***_ is “individual time varying error distributed independently”. For computation of ϴ, some specific approach is needed because ϴ _***i***_ and ϴ _***t***_ are related to reforms in many non-determined sources so Eq (1) including control variable turns, where YP is per capita GDP;

$$EP_{it}={ϴ}_{i}+{ϴ}_{t}+ϴREF_{it}+ϴYP_{it}+\epsilon_{it}$$ (2)

If ϴ _***i***_ and ϴ _***t***_ are dependent on reforms, then first difference may be taken for estimation so Eq (2) becomes;

$$\Delta_{t}EP_{it=}\Delta_{t}{ϴ}_{t}+ϴ\Delta_{t}REF_{it}+ϴ\Delta_{t}{\mathrm{YP}}_{it}+\Delta_{t}\varepsilon_{it}$$ (3)

“Where Δ_***t***_ is difference of individual observations across periods and Δ _***t***_ ϴ_***t***_ is difference in common time effects. But there are two periods in the model; pre reforms and post reforms period. Difference in differences estimator takes the difference between the differences between the two groups such that:

$$B=\{E(EP_{i1}{}^{t}\;l\;REF_{i1})‐E(EP_{i1}{}^{t}\;l\;REF_{i0})\}–\{E(EP_{i0}{}^{c}\;l\;REF_{i1})‐E(EP_{i0}{}^{c}\;l\;REF_{i0})\}$$ (4)

Superscript *t* and *c* in Eq (4) represent the treated and control groups respectively, ***E(EP***_***i1***_^***t***^ ***l REF***_***i1***_***)*** is expected outcome of countries after reforms while ***E(EP***_***i1***_^***t***^ ***l REF***_***i0***_***)*** is outcome of same group before reforms. In the same way**, *E(EP***_***i0***_^***c***^ ***l REF***_***i1***_***)*** is outcome of control after reforms in treated group and ***E(EP***_***i0***_^***c***^ ***l REF***_***i0***_) is outcome of control group before the reforms. Two structural assumptions are mandatory for difference in difference estimation. One is common time effect across the control and treated groups while other is stable composition of both groups before and after reforms” [45]. Upon violations of these assumptions, Giavazzi and Tabellini [22] described many possibilities to decrease the violations of these assumptions; “First, include in the control variables dummies to capture the characteristics that make countries different. The second suggestion is to include in the control group both countries that have not experienced reform at all and countries that have experienced reform before the beginning of the sample period.”

There are many advantages of DID approach, especially when pre and post policy effects have to be analyzed [46]. DID is a microeconomic approach that handles many critical endogeneity issues when comparing two heterogeneous individuals. The treatment effect can be measured from treated and control group over time. Moreover, this method permits to estimate the variations within and outside the country [47]. The treated and control group may be compared before and after policy implications.

## 3. Data and its sources

This study used the “Environmental Performance Index” (EPI) to gauge the environmental performance of economies in account of humans’ protection from environmental harms and protection of eco system. There are two main weighed indicators in the index: “Ecosystem Vitality (70%) and Environmental Health (30%), is divided into 10 policy categories, overall measuring 22 different indicators. EPI is a positive indicator, meaning that the higher the EPI, the better the respective country’s environmental performance. EPI succeeds in combining many indicators—which were only individually taken into account when testing environmental quality—in one. It is becoming quite popular in measuring environmental performance due to its integration of academic research, thus making it, in the authors’ opinion, the most complete and appropriate indicator for the overall measurement of environmental performance” [48].

There are two broad categories of institutions: political and economic institutions. Economic reforms are defined as comprehensive and large alterations to advance regulatory quality, rendering monetary and fiscal institutions’ independence, protecting property rights, reducing corruption, strengthening of judiciary, and enhancing corporate governance. The opportunities are created for people through these reforms for their participation in economic activities. The quality of economic institutions is measured through the economic freedom index obtained from “The Heritage Foundation”. To measure the “economic freedom index”, 12 quantitative and qualitative variables are divided into four sub-categories; regulatory efficiency, government size, rule of law, and open markets.

Political institutions are “political rules of the game”. These are constraints and regulation governing political processes and decisions making along with ability of citizens to meet the objectives of that process. Political reforms are comprehensive modification connected with how power is constituted and practiced. POLITY IV is used to measure the political institutions ranging from -10 to +10 reflecting hereditary monarchy to consolidated democracy.

The criteria for political and economic reforms are taken from [22, 49]. Economic reforms are calculated using forward and backward moving average. “The economic reforms are considered in those countries where forward moving average is greater than backward average by at least 12 points. The reforms are divided into two heads; big and small reforms. If forward moving average is greater by at least 2 points, then it is considered as small reforms but if it is greater than by at least 4 points then it is considered as big reforms. The political institutions reforms are considered when a country crosses the Polity Scores above zero because zero value shows the end of autocracy. So the non-negative value of a country is considered as a treated group while zero value is treated as a control group.” Table 1 describes the details of each variable.

**Table 1:** Variables and their description.

Variables	Descriptions
ECR	1 if economic reforms occur from the year, if not then 0
BECR	1 if big economic reform occur from the year, if not then 0
SECR	1 if small economic reforms occur from the year, if not then 0
PLR	1 if political reforms occur from the year, if not then 0
TPREC	1 if there are 3 years preceding economic reforms, if not then 0
TPRPL	1 if there are 3 years preceding political reforms, if not then 0
TPSEC	1 if economic reforms start in the year and remain for 3 years, if not then 0
TPSPL	1 if political reforms start in the year and remain for 3 years, if not then 0
FBYPL	1 if political reforms are in 4^th^ year and beyond, if not then 0
ECPL	1 if country reforms economic institutions before political, if not then 0
PLEC	1 if country reforms political institutions before economic, if not then 0

GDP per capita is gained from the “World Development Indicators”. All the data is gathered from 1996–2020 for middle and lower income economies categorized by the “World Bank”. The sample and time period is selected because of restrictions in available data. All selected economies have similar institutional structure and are labelled as developing countries.

## 4. Empirical findings and discussion

Difference in difference (DID) technique is regressed to determine the relation between institutional reforms and environmental performance and results are pasted in the following Tables 2–4.

**Table 2:** Impact of political reforms on environmental performance.

	Environmental Performance	
Variable	Model I	Model II
**Constant**	1.33*** (0.648)	2.49***(1.152)
**PLR**	0.171**(0.058)	
**TPRPL**		0.049 (0.051)
**TPSPL**		0.051** (0.044)
**FBYPL**		0.286* (0.047)
**YP**	0.529** (0.724)	0.821* (1.522)
**R** ^**2**^	0.028	0.035

Note: The sign *, ** and *** show significance at 1%, 5% and 10% respectively. Bootstrap robust standard errors are in parentheses.

**Table 3:** Impact of economic reforms on environmental performance.

	Environmental Performance		
Variables	Model-I	Model-II	Model-III
**C**	0.651 (4.77)	7.482*** (3.914)	13.27*** (4.614)
**BECR**	0.214*** (0.046)		
**SECR**		0.371** (0.062)	
**TPREC**			-0.019 (0.037)
**TPSEC**			0.017* (0.029)
**YP**	0.271** (0.381)	-0.392*** (0.183)	0.416*** (0.847)
**R-squared**	0.061	0.522	0.038

Note: The sign *, ** and *** show significance at 1%, 5%, and 10% respectively. Bootstrap robust standard errors are in parentheses.

**Table 4:** Impact of economic and political reforms on environmental performance.

	Environmental Performance
**Constant**	0.928* (0.712)
**ECR**	0.139**(0.128)
**PLR**	0.161** (0.057)
**ECPL**	0.274*** (0.006)
**PLEC**	0.181*** (0.014)
**R-squared**	0.035

Note: The sign *, ** and *** show significance at 1%, 5% and 10% respectively. Bootstrap robust standard errors are in parentheses.

The empirical results describing the relationship between environmental performance and political reforms are reported in the above Table 2. The findings reveal that a country’s environmental performance increases also as political reforms occur and the relationship holds afterwards, i.e., that environmental performance increases as political reforms prevail even after three and four years of political reforms. This implies that political reforms provide the fundamental conditions for environmental performance because people are involved in decision making demanding better health and environmental living conditions [50]. This really amalgamates political institutions with market economy and represents the critical role for environmental performance in developing countries. It is found that 3 years before political reforms do not contribute significantly to improve the environmental performance. Three years post political reforms and beyond, reforms positively correlate with environmental performance as well, overall suggesting that political reforms positively affect environmental performance. The relevant literature suggests that the political reforms have crucial importance for developing economies through raising the level of FDI and liberalization of capital and financial markets, and an open economy assists to protect the environment [51, 52]. There is no immediate effect of political reforms on the countries but it is a gradual and slower process to have their positive impact [53, 54]. Frankel and Rose [55] also found the correlations among GDP, environmental regulations, democracy, environmental quality, and trade. Their findings reveal that free democratic institutions authorize their people to demand good environmental regulations and regulatory regimes to increase the environmental quality. In the same way, Frazin and Bond [56] identified that freedom and democracy are essential to freely express the preferences of economic agents for environmental quality. It is also evident that in the beginning, political reforms create uncertainty in a society but then trust in political institutions is restored and investors have more attraction for investment, leading to spread of green technology and the economy improves its environmental performance [47]. The per capita income also increases due to political reforms by improving environmental performance as many studies [27–29, 45, 47, 53, 55] are of the view that exports of democratic economies increase along with increase in economic activities, so rising per capita income. The well planned economic and political structure may revolutionize the environmental performance as findings of the studies [57, 58] highlight that democratic countries have more macro-economic stability.

In the above Table 3, the effects of economic reforms are analyzed for environmental performance. There are two categories of economic reforms; small and big reforms. The computed coefficients show the mean performance of treated group as compared with control group, revealing that economic reforms improve the environmental performance. It is evident that post reforms in 3 years are crucial to protect the environment. The countries with small reforms also contribute positively for environmental performance. [39, 40]. In addition to this, more than three years of economic reforms are mandatory to increase environmental performance because post three years’ reforms alter the economic structure and firms are encouraged to use environment friendly techniques for production. Even small economic reforms enhance the level of environmental performance while big economic reforms are strongly associated with environmental performance [42]. The impacts of post reforms on environmental performance are determined and empirical findings reveal that economic reforms sustain the environmental quality only when it improves continuously for more than 3 years. If societies reform the economic institutions continuously then environmental performance improves. The economies remain dependent on small reforms but do not move toward big reforms, are not able to achieve higher levels of environmental performance and even become negative after a while. Moreover, big reforms carry environmental friendly policies and high economic freedoms, sustaining and boosting economic growth at a higher rate. The empirical outcomes of the study are in line with [28, 29]. The studies like [14, 20, 21, 33] depict the positive effect of economic institutions on economic growth. Moreover, economic growth associated with economic reforms enhance environmental performance. It can be argued that higher economic growth is a source to protect the environment as rich countries have large numbers of educated people demanding better and healthy living conditions so there are well established environmental standards for industry.

The findings in context of interaction between economic and political reforms are reported in above Table 4, there are interesting findings. It is found that one type of reforms leads to other type of reforms; means political reforms stimulate economic reforms and vice versa. Moreover, each type of reform positively affects the environmental performance in developing countries. The study [40] investigated the effect of economic reforms on political reforms and vice versa and found that each type of reform triggered the other. The same outcomes are supported by many studies [23, 42, 45, 51]. Economic reforms are a source stabilizing the financial market, the trust of investors and people restores if any type of reforms prevail in an economy so green technology will flourish the economy. The findings of the studies [8, 9, 14–16, 19, 59, 60] convey that institutions have crucial importance for environmental performance. Based on the findings of the study, it is highlighted that economic and political reforms are both crucial for environmental protection in developing countries. The environment may be protected significantly through market mechanisms and political structure. The political reforms frame the rules for environmental protection while economic reforms help the production sector to be more environment friendly. The inefficient institutions and bad governance are associated with environmental degradation.

## 5. Conclusions

Since 1992, “United Nations Framework Convention on Climate Change” has been established to improve the quality of air by decreasing the quantity of air pollutants like Carbon Dioxide emission and then actively pursued as a global agenda. All the members agreed to reduce the air pollutants to overcome the issue of global warming and climatic changes. The combating of environmental performance remained a hot and important topic among researchers and policy makers [61]. Many countries adopted multiple policy measures to protect the environment but the outcomes of these policy measures varied from region to region [62]. However, the impact of institutional reforms on environmental protection remained unknown in the existing literature. The findings of the study highlighted the institutional reforms as an important driver of environmental protection in developing countries. Environmental problems affecting developing countries are not because of technological failings only but also institutional failings. Ever increasing challenges are demanding the efficient implementations of institutional reforms nowadays. Requirement of development collaborators, changing in global terms of trade, and internal and external pressures are the reasons to trigger the reforms. These reforms are a source to provide a fair profit return and less risky environment having attraction for investors, increasing environmental performance as well as economic growth. The investors require a less risky environment for investing their money.

It was hypothesized that institutional reforms positively affect the environmental performance in developing countries. The purpose was to investigate the importance of institutional reforms in the area of environmental protection and sustainability. So this paper attempted to explore the relation between institutional reforms and environmental performance through a novel way by segregating the political and economic institutional reforms. The macro level variables and environmental performance index are used to explore the impacts of reforms on environmental performance in 122 developing economies for the period from 1996–2020 by applying difference in difference (DID) approach. Though the environment and institutions have been suggested to affect each other but the relationship between institutional reforms and environmental performance has not been examined. The findings show that the environmental performance index has positive correlation with economic and political institutional reforms. This provided a sign that an economy’s environmental performance increases as with higher levels of institutional reforms. Many studies provided theoretical or empirical confirmations consistent with few conclusions of this study or gave a handsome explanation of some conceptual connection of this study’s findings.

It is beneficial to state that the relation between environmental performance and institutional reforms can be elaborated by the fact that institutional reforms provide a rich ground to protect the environment in developing countries. Moreover, longevity of institutional reforms in any country has prime importance to explain the environmental performance. It is found that political reforms are a source to increase the level of environmental protection. When democracy in a country prevails then people have more rights as compared with non-democratic countries. So people in democratic countries are free to express their thoughts and opinions. These people demand a pollution free environment for their own and future generations from the ruling authorities [63–66]. The findings of the earlier literature reveal that democratic economies have stricter rules in favor of environmental protection. This study is also an addition in literature by establishing a relationship among political reforms, economic reforms and environmental performance because reforms drive to change the behaviors of economic agents to be more environmental friendly. So this study broadened the cluster of institutional variables by considering economic and political variables for a better explanation of environmental performance.

However, this study has some limitations that may be helpful for future research. Though the indices of Environmental Performance Index are reliable and follow the standard statistical procedures, environmental performance may be measured by combining some other variables of environment. It would have value for future exploration to recognize an econometric model with many factors, apart from economic growth, that may affect environmental performance.
